The article "CD4-Targeted T Cells Rapidly Induce Remissions in Mice with T Cell Lymphoma" was retracted in 2024. Reasons: signs of a paper mill; suspected computer-generated content; unreliable results or conclusions; concerns about the data.

# CD4-Targeted T Cells Rapidly Induce Remissions in Mice with T Cell Lymphoma

**DOI:** 10.1155/2021/6614784

**Published:** 2021-03-27

**Authors:** Jie Cheng, Guanghua Chen, Hui Lv, Liangjing XU, Huiwen LIU, Tianping Chen, Lijun Qu, Jian Wang, Lemei Cheng, Shaoyan Hu, Yi Wang

**Affiliations:** ^1^Department of Hematology, Children's Hospital of Soochow University, Suzhou, Jiangsu Province, China; ^2^Department of Hematology, Anhui Provincial Children's Hospital, Anhui Province, China; ^3^Jiangsu Institute of Hematology, The First Affiliated Hospital of Soochow University, Suzhou Jiangsu Province, China

## Abstract

**Objective:**

To explore the immune cell therapy for T cell lymphoma, we developed CD4-specific chimeric antigen receptor- (CAR-) engineered T cells (CD4CART), and the cytotoxic effects of CD4CART cells were determined in vitro and in vivo.

**Methods:**

CD4CART cells were obtained by transduction of lentiviral vector encoding a single-chain antibody fragment (scFv) specific for CD4 antigen, costimulatory factor CD28 fragment, and intracellular signal transduction domain of CD3 fragments. Control T cells were obtained by transduction of reporter lentiviral vector. The cytotoxicity, tumor growth, and survival rate of mice with T cell lymphoma were analyzed after adoptive T cell transfer in vivo.

**Results:**

CD4CART cells had potent cytotoxic activity against CD4+ T1301 tumor T cells in a concentration-dependent manner. In addition, adoptive CD4CART cell transfer significantly suppressed tumor growth and improved animal survival with T cell lymphoma, compared to the mice who received control T cells and PBS.

**Conclusion:**

CD4CART cells have potent cytotoxic effects on T cell lymphoma. The study provided an experimental basis for CD4CART-mediated therapy of T cell lymphoma.

## 1. Introduction

T cell lymphoma is a rare form of cancerous lymphoma affecting T cells and patients with cutaneous T cell lymphoma (CTCL) are at a higher risk of developing second malignancies [1]. There is no effective treatment for this debilitating disease so far. Anti-PD-1 and anti-CTLA-4 antibodies have been recently developed as checkpoint reagents in the treatment of various cancer patients including Hodgkin lymphoma and showing some promising results in clinical trials [2–4]. Other reagents, such as TIM-3, TIGIT, BTLA, CD47, and KIR that target the adaptive and innate immune system are recently developed as alternative ways to activate the immune system [5]. However, the results were elusive among patients with non-Hodgkin lymphomas.

T cell-mediated therapy against cancer was developed in 2003 by Dr. Rosenberg through amplification and adoptive transfer of tumor-infiltrating lymphocytes (TILs) in the patients; the therapeutics have been confirmed great success in patients with melanoma [6, 7]. Because the number of TILs from patients is limited and the expansion of TILs in vitro is difficult, a novel T cell therapy approach was developed recently, by which naive T cells were modified to express chimeric T cell antigen receptor (CAR) encoding tumor-associated antigen- (TAA-) specific single-chain antibody fragment (scFv) and intracellular domain of CD3zeta [8–10]. After the cognate CAR-T cells were administered into cancer patients, the adoptively transferred T cells can migrate into tumor sites by specifically binding to TAA on cancer cells. A body of evidence confirmed that CAR-T cells have longer survival ability and more cytotoxic effects in vivo with intracellular activation domains, 4-1BB and CD3zeta [11, 12]. Recently, CD19-targeted CAR-T cell therapy has been successfully explored in clinical trial and showed an overall response rate of 67% without obvious side effects [13–17]. Because B cells exclusively express high levels of CD19 cell surface molecule, which makes it an ideal target in CD19-targeted CAR-T cell therapy. Because T cell lymphoma is only 10-15% of non-Hodgkin's lymphoma, the research on CAR-T-mediated therapy for T cell lymphoma is well investigated. Though a study on CD1a-targeted CAR-T for T cell acute lymphoblastic leukemia (T-ALL) was reported, the therapeutic effects were still elusive [18]. Thus, it is urgently required to develop an effective approach in the treatment of T cell lymphoma.

The article "CD4-Targeted T Cells Rapidly Induce Remissions in Mice with T Cell Lymphoma" was retracted in 2024. Reasons: signs of a paper mill; suspected computer-generated content; unreliable results or conclusions; concerns about the data.

Because CD4 antigen is present in the most of T cell lymphoma and some T lymphocytic leukemia cells [19], but it is not highly expressed in hematopoietic stem cells and non-hematopoietic cells, the property makes CD4 antigen as an ideal target in CAR-T cell therapy against T cell lymphoma and some T lymphocytic leukemia [20]. A body of evidence showed that monoclonal anti-CD4 antibody was effective in the treatment of some autoimmune diseases in animal models and clinical trials without obvious side effects [21–23]. Therefore, CD4-targeted immune cell therapy may be a promising therapeutic approach in the treatment of T cell lymphoma without obvious side effects. To explore the possibility of CD4 antigen-targeted CAR-T cell therapy, we in this study engineered CD4-target T cells (CD4CART), and antitumor activity was determined in vitro and in vivo.

## 2. Materials and Methods

### 2.1. Construction of Lentiviral Vectors

A CD4-CAR fusion protein fragment containing a single-chain antibody fragment (scFv) specific for CD4 antigen, costimulatory factor CD28 fragment, and intracellular signal transduction domain of CD3 fragments was constructed into pGIPZ transfer vector (Cat. TLP4614, Open biosystems, Huntsville, AL, USA, Figure 1(a)). The correct insert and DNA sequence in the plasmid were confirmed by enzyme digestion. The control reporter plasmid pRL Renilla luciferase reporter pRL-CMV vector (Cat. E2261, Promega, Madison, WI, USA) was used as controls. The fusion protein expression was further determined by Western blot analysis after transfer into 293T cells. The transfer recombinant plasmid was then engineered into lentiviral vector Lv.CD4-CAR by cotransfection of 293T viral packaging cells with this plasmid and other packaging plasmids (pTLA1-Pak, pTLA1-Enz, pTLA1-Env, pTLA1-Rev). 2 days after plasmids cotransfection, the conditional media of the transfected cells containing lentiviral vector Lv.CD4-CAR were collected and virus titer was determined in 293T cells and virus stock was frozen in -80°C freezer.

The article "CD4-Targeted T Cells Rapidly Induce Remissions in Mice with T Cell Lymphoma" was retracted in 2024. Reasons: signs of a paper mill; suspected computer-generated content; unreliable results or conclusions; concerns about the data.

### 2.2. Lentivirus Transduction of T Cells

After lentiviral titer was determined, CD4+ T cells purified from peripheral blood in 6-well plate were incubated with anti-CD3 and anti-CD28 antibodies (Cat. 16-0037-81, 16-0289-81, eBioscience, San Diego, CA) to activate the naive T cells to improve lentiviral vector transduction efficiency, according to the previous report [12]. 24 hours after cell activation, the activated T cells were infected with the lentiviral vector at multiplicity of infection (MOI = 10) for 48 hours to obtain the engineered T cells expressing CD4-CAR on cell surface (CD4CART). The viral vector transduction efficiency was measured by protein L binding activity (Cat. ab155706, Abcam, Cambridge, MA). Because protein L can bind to the kappa light chain of scFv in chimeric antigen receptor (CAR) [24], protein L becomes an ideal reagent in the detection of CAR expression in the CD4-CAR-transduced T cells. A high protein L binding activity reflects a high expression level of CD4-CAR on CD4CART cells. Finally, the engineered T cells were maintained and expanded in RPMI1640 culture media for 7 days before cell adoptive transfer.

### 2.3. CD4CART Cytotoxicity Assay In Vitro

After 7 days of expansion, the cytotoxic activity of CD4CART cells or control T cells on tumor cells was confirmed by incubation with T lymphoma cell line, CD4+ T1301 cells (Cat. 01051619-CDNA, Merck, Kenilworth, NJ) at a ratio of 0 : 1, 0.5 : 1, 1 : 1, 2 : 1, 4 : 1, and 8 : 1. After 24 hours of coculture and staining with anti-CD3 and anti-CD4 antibodies (Cat. 357407, 300307, Biolegend, San Diego, CA), the depletion of CD4+ targeted tumor cells were analyzed by flow cytometry analysis.

### 2.4. CD4CART Cytotoxicity Assay In Vivo

8-12 years old of male immune-deficient NSG mice (The Jackson Laboratory, Bar Harbor, Maine) were subcutaneously (s.c.) injected with 4 × 10^6^ CD4+ T1301 tumor cells to establish a mouse model with T cell lymphoma. All animal experiments were approved by the Committee of Animal Care and performed in the animal facility of Nanjing University of Medical School in China. 1 week after tumor cell inoculation, 1 × 10^6^ CD4CART single-cell suspension in 0.7 ml volume was intravenously administered into the mouse model. Meanwhile, the mouse model received the same doses of naive T cells or PBS was administered as untreated control group. Tumor size and mouse survival were recorded every other day.

The article "CD4-Targeted T Cells Rapidly Induce Remissions in Mice with T Cell Lymphoma" was retracted in 2024. Reasons: signs of a paper mill; suspected computer-generated content; unreliable results or conclusions; concerns about the data.

## 3. Results

### 3.1. Generation of CD4CART Cells

Recombinant transgene plasmid pCD4-CAR containing a single-chain antibody fragment (scFv) specific for CD4 antigen, costimulatory factor CD28 fragment, and intracellular signal transduction domain of CD3 fragments was constructed by molecular cloning as shown in diagram of Figure 1(a). The correct insert in the recombinant plasmid was confirmed by EcoRI and BamHI digestion. After agarose gel electrophoresis, we observed a 1.5 kb band, indicating the presence of insert gene fragment, whereas null plasmid without insert did not contain the insert (Figure 1(b)). Lentiviral vector Lv.CD4-CAR containing CD4-CAR was generated by cotransfection of transgene plasmid pCD4-CAR and other packaging plasmids into 293T packaging cells. The conditional media of transfected cells containing lentiviral vector Lv.CD4-CAR were collected. The viral titer was measured in HeLa cells with serial dilution of viral vector. The unconcentrated viral titers were at a range of 0.8 − 1.0 × 10^6^ transducing units/ml (TU/ml).

To modify T cells with CD4-CAR, the naive T cells were infected with Lv.CD4-CAR at multiplicity of infection (MOI) of 10 for 2 days. The engineered T cells were maintained and expanded in RPMI1640 culture media for 7 days. The CD4-CAR expression level on engineered CD4CART cells was determined by measuring protein L binding activity to kappa light chain of scFv on CD4CART cells. We observed that the protein L binding activity to CD4CART cells was as high as 47.5%, whereas the protein L binding activity to control T cells was only 2% (Figure 1(c)), indicating the high expression level of CD4-CAR on the modified T cells. Additionally, we also observed that CD4+ T subset was almost completely depleted 3-4 days following Lv.CD4-CAR transduction. However, the control T cells had the normal proportion of CD4+ T cells (Figure 2). The data indicated that CD4CART cells exhibit potent anti-CD4 activity in vitro.

### 3.2. CD4CART Cells Exhibited Potent Cytotoxic Activity In Vitro

To investigate the role of CD4CART cells in antitumor cell activity, we coincubated the CD4CART cells (effector cells, E) with CD4+ T1301 tumor cells, a T-ALL cell lines (target cells, T) at different E : T ratio. 24 hours after coculture, we observed a more reduced population of CD4+ T1301 tumor cells at an E : T ratio of 4 : 1 than the ratio at 2 : 1. However, the control T cells did not exhibit cytotoxic activity against CD4+ T1301 tumor cells (Figures 3(a) and 3(b)).

The article "CD4-Targeted T Cells Rapidly Induce Remissions in Mice with T Cell Lymphoma" was retracted in 2024. Reasons: signs of a paper mill; suspected computer-generated content; unreliable results or conclusions; concerns about the data.

### 3.3. CD4CART Cells Exhibited Potent Cytotoxic Activity in Mice with T Cell Lymphoma

To evaluate in vivo antitumor activity of CD4CART cells, we developed a xenogeneic mouse model. Mice with lymphoma tumor were established by subcutaneously (s.c.) injection with 4 × 10^6^ CD4+ T1301 tumor cells at armpit of 6-8 weeks old NSG mice. 1 week after tumor cell inoculation, 1 × 10^6^ CD4CART single cells were intravenously administered into the tumor site of mouse model. Mice treated with the control T cells or PBS were as the untreated controls. 15 days after the treatment, we observed the slower tumor growth in the mice who received CD4CART cells (Group: CD4CART cells) than the mice who received the same doses of naive control T cells (Group: T cells) or PBS (Group: PBS) (Figure 2(a)). Quantitative analysis showed that the tumor size in CD4CART group was significantly smaller than the mice in both naive control T cell group and PBS control group (*p* < 0.001, *n* = 10). The mice treated with control T cells and PBS had an average tumor size of 80 mm^3^ on day 17 posttumor cell inoculation (Figure 2(b)). However, the tumor size glowed very slowly in the mice treated with CD4CART cells, and 2 mice had disappeared tumor 30 days after the treatment.

### 3.4. CD4CART Cells Increased Survival of Mice with Lymphoma Tumor

Our further analysis showed that CD4CART cells significantly improved the survival of mice with T cell lymphoma. We observed 3 mice died, respectively, on day 15, 23, and 30 after CD4CART cell treatment, and other mice remained healthy and survived until the end of the experiments on day 50. The survival rate reached up to 50%. However, 6 mice died on day 13, 18, 20, 21, 24, and 25, respectively, after the treatment with control T cells. 6 mice died on day 12, 20, 21, 21, 23, and 24, respectively, after treatment with PBS. All mice received control T cells and PBS died at the end of the experiment. The survival rate was comparable between mice treated with control T cells and PBS (*p* > 0.05, *n* = 10). Therefore, CD4CART cell treatment significantly improved the survival rate of mice, compared to the treatment with control T cells and PBS (*p* < 0.001, *n* = 10) (Figure 2(c)).

The article "CD4-Targeted T Cells Rapidly Induce Remissions in Mice with T Cell Lymphoma" was retracted in 2024. Reasons: signs of a paper mill; suspected computer-generated content; unreliable results or conclusions; concerns about the data.

## 4. Discussion

T cell lymphoma is a rare form of cancerous lymphoma affecting T cells, which represents less than 15% of all non-Hodgkin's diseases. Various risk factors and virus infections such as Epstein Barr virus and human T cell leukemia virus-1 account for the progression of T cell lymphoma [25, 26]. Unfortunately, there is no effective therapeutics for the debilitating disease so far. Cell-based therapy, particularly CAR-T cell therapy, has been confirmed effective in some B cell lymphatic diseases, such as B cell leukemia. However, CAR-T cell therapy for T cell lymphoma is not well developed so far. In this study, we explored a novel therapeutic approach in the treatment of murine T cell lymphoma by CAR-T adoptive cell transfer, in which a single-chain antibody fragment (scFv) specific for tumor-associated antigen CD4 was engineered into naive CD4+ T cells. To improve the modified T cell antitumor activity, scFv fragment was fused with costimulatory factor CD28 fragment and intracellular signal transduction domain of CD3 fragments [12]. Our results in vitro demonstrated that CD4 scFv-engineered T cells had potent cytotoxic effects on CD4+ T1301 tumor cells, a T-ALL cell lines at a concentration-dependent manner. The tumor cell viability was significantly reduced starting at E : T ratio of 0.5 : 1. The effects were further confirmed in tumor animal model, in which mice treated with CD4CART cells had much slower tumor growth and higher survival rate than the mice who received control T cells and PBS. We observed 3 death and 2 mice without tumor growth in the CD4CART, which reached the total survival rate up to 50% at the end of the experiment. However, all mice received the treatment with control T cells and PBS died at the end of the experiment. The results provided solid evidence that CD4CART cells were potent in the treatment of mice with T cell lymphoma.

In addition, we did not observe the side effects of CD4CART cell infusion in vivo. We speculate that the low side effects may be caused by high expression of CD4 in T cell lymphoma but low expression in hematopoietic stem cells and normal CD4+ T cells. The concepts were also supported by previous studies showing that administration of monoclonal antibody against CD4 did not elicit significant side effects in autoimmune diseases, such as psoriasis [21] and multiple sclerosis [22, 23]. There are no reports so far about significant depletion of normal CD4+ T cells and suppression of immune system after anti-CD4 antibody treatment in animal model. Given that the population of normal CD4+ T cells is reduced after anti-CD4 antibody treatment [27], new normal CD4+ T cells should be effectively produced and expanded in bone marrow, and the number is gradually increased after monoclonal antibody treatment. Therefore, CD4+ normal T cells were reversible in vivo. CD4-targeted therapy is safe and effective in the treatment of T cell lymphoma. The survival, dynamics, and side effects of CD4CART cells will be further evaluated in the future.

The article "CD4-Targeted T Cells Rapidly Induce Remissions in Mice with T Cell Lymphoma" was retracted in 2024. Reasons: signs of a paper mill; suspected computer-generated content; unreliable results or conclusions; concerns about the data.

## 5. Conclusion

In this study, we generated CD4-targeted T cell therapy for T cell lymphoma. The study in vitro and in vivo confirmed that CD4CART cells were potent in defense against T cell lymphoma without significant side effects. The study provided a novel therapeutic approach in the treatment of T cell lymphoma.

## Figures and Tables

**Figure 1:** Generation of CD4-CAR-T cells. (a) Diagram of recombinant plasmid pCD4-CAR containing a single-chain antibody fragment (scFv) specific for CD4 antigen, costimulatory factor CD28 fragment, and intracellular signal transduction domain of CD3 fragments. H indicates hinge region; TM indicates transmembrane region. (b) Identification of correct transgene insert by enzyme digestion and electrophoresis. Plasmid was digested with EcoRI and BamHI. 1.5 kb band indicates insert fragment and 8.6 kb band indicates vector backbone. (c) Flow cytometry analysis for the CD4-CAR modified T cells after Lv.CD4-CAR vector transduction. The positive engineered T cells were analyzed by measuring protein L binding activity to kappa light chain of scFv on CD4-CAR-T cells. Control indicated that T cells were infected with null reporter vector expressing luciferase.

**Figure 2:** CD4-CAR-T cells increased survival of mice with T cell lymphoma. Mouse model with T cell lymphoma was established by subcutaneously (s.c.) injection with 4 × 10^6^ CD4+ T1301 tumor cells. 1 week after tumor cell inoculation, the mice were received treatment of 1 × 10^6^ CD4CART cells (CD4CART group), control T cells (T cell group), or PBS were intravenously (i.v.). (a) Tumor size of the treated mouse was viewed by fluorescence stereomicroscope. Representative photograph of one mouse in each group. (b) Quantitative analysis of tumor size in each group, *n* = 10, ^∗∗^*p* < 0.001, vs. the CD4CART group. (c) Survival rate of mice in each group after treatment.

**Figure 3:** CD4-CAR-T cells exhibited potent cytotoxic activity in vitro. The cytotoxic activity of CD4-CAR-T cells was determined by coculture of CD4-CAR-T cells or control T cells (effector cells, E) with T1301 tumor cells, a T-ALL cell lines (target cells, T) at different E : T ratio. CD4+ and CD8+ T cells were analyzed 24 hours after coculture by flow cytometry analysis. (a) Representative plot was shown for each treatment. (b) Quantitative analysis of cytotoxic activity of CD4-CAR-T cells at different E : T ratio. Data was presented as mean ± standard error, *n* = 3, ^∗∗^*p* < 0.001, vs. T cell group.

The article "CD4-Targeted T Cells Rapidly Induce Remissions in Mice with T Cell Lymphoma" was retracted in 2024. Reasons: signs of a paper mill; suspected computer-generated content; unreliable results or conclusions; concerns about the data.

## Data Availability

Some or all data, models, or code generated or used during the study are available from the corresponding author by request.
